RETRACTED

# Effect of Intelligent Medical Management Platform Combined with Perioperative Detailed Nursing on Cognitive Ability, Postoperative Complications, and Quality of Life of Patients Undergoing Hysterectomy

**DOI:** 10.1155/2022/4820835

**Published:** 2022-04-16

**Authors:** Xiaodao Han, Meng Zhang, Shanshan Jiang, Chunni Hao

**Affiliations:** ^1^Day Chemotherapy Ward, Qingdao Central Hospital, 266000 Qingdao City, Shandong Province, China; ^2^Department of Critical Medicine, Qingdao Central Hospital, 266000 Qingdao City, Shandong Province, China; ^3^Gynecological Oncology, Qingdao Central Hospital, 266000 Qingdao City, Shandong Province, China; ^4^Medical Record Management Department, Yantaishan Hospital, Yantai City, Shandong Province, China

## Abstract

**Objective:**

To analyze the effect of an intelligent medical management platform combined with perioperative detailed nursing on cognitive ability, postoperative complications, and quality of life (QOL) of patients undergoing hysterectomy.

**Methods:**

The clinical data of 76 patients undergoing hysterectomy in our hospital from December 2019 to December 2021 were selected for the retrospective analysis, and the patients were divided into the experimental group (EG, *n* = 38, intelligent medical management platform+perioperative detailed nursing) and the routine group (RG, *n* = 38, routine nursing) according to their admission order, and the cognition of disease and QOL after intervention of patients in the two groups were evaluated by the self-proposed questionnaire on cognition of disease of our hospital and the MOS 36-item short-form health survey (SF-36).

**Results:**

After intervention, the scores on cognitive ability, various nursing items, and QOL were significantly higher in EG than in RG (*P* < 0.001), and during the study, the total incidence rate of complications was significantly lower in EG than in RG (*P* < 0.05).

**Conclusion:**

Combining an intelligent medical management platform with perioperative detailed nursing is a reliable method to improve QOL and reduce postoperative complications for patients undergoing hysterectomy. Further research will be conducive to providing a reliable perioperative intervention scheme for such patients.

## 1. Introduction

Hysterectomy is a common gynecological surgical procedure, and its indications include benign uterine tumors, malignant tumors of the ovary or fallopian tube, uterine rupture, and uterine prolapse [1]. Its surgical trauma is large, which can easily lead to postoperative stress incontinence, vaginal relaxation, insomnia, and other problems in patients, adversely affecting patients' postoperative quality of life (QOL) and family function [2, 3]. Routine perioperative nursing often leads to poor intervention outcomes due to the more single measures [4]. Detailed nursing, however, adheres to the concept of person-centered services, which greatly improves the clinical nursing effect with the measures such as preoperative nursing, diet intervention, and medication guidance included, and such a nursing model puts the patients' nursing needs in the first place, thereby greatly enhancing the quality of nursing and realizing the humanization of nursing while increasing the degree of satisfaction with clinical nursing. The effect of detailed nursing has been demonstrated in patient population with lung cancer, coronary heart disease in the elderly with type 2 diabetes, and other diseases [5, 6]. With the advancement of big data era, intelligent medical tools with the advantages of real-time review and long-time preservation are widely used in the clinical management of hospitalized patients and have now been used in patient populations such as those with lumbar degenerative diseases and young and middle-aged hypertension [7, 8]. In this study, with the help of an intelligent medical tool, nursing intervention was implemented for patients undergoing hysterectomy throughout the whole process from patient admission to postoperative rehabilitation, in the hope of providing better perioperative nursing services for such patients and then effectively improving prognosis, which is of great significance to improve patients' postoperative QOL and reduce the occurrence of complications. The results are reported as follows.

RETRACTED

## 2. Material and Methods

### 2.1. General Data

The study subjects were 76 patients undergoing hysterectomy in our hospital from December 2019 to December 2021, and the study met the World Medical Association Declaration of Helsinki (2013) [9]. The patients were divided into the experimental group (EG) and the routine group (RG) according to the admission order. The inclusion criteria were as follows. (1) The patients had stable vital signs and needed hysterectomy upon diagnosis; (2) the patients fully understood the intervention plan; and (3) the patients were 18-75 years old. The exclusion criteria were as follows. (1) The patients had fluid and electrolyte imbalance and coagulation dysfunction; (2) the patients were complicated with cervical cancer or other severe gynecological diseases; and (3) the patients had diseases in the liver, heart, kidney, and other organs.

### 2.2. Methods

After admission, all patients received routine examinations to measure their body temperature, blood glucose, blood pressure, etc. [10], and accepted the hysterectomy. Patients in RG received clinical routine nursing during the perioperative period including the following steps: conducting education of clinical basic knowledge, keeping the wards tidy and clean, regularly replacing bed sheets, quilt covers, and pillow towels for the patients, and informing the patients of relevant precautions such as diet and exercises before surgery [11, 12].

RETRACTED

Patients in EG received an intelligent medical management platform combined with perioperative detailed nursing with the following specific steps:

1. Perioperative detailed nursing. ① Preoperative nursing: the patients were repeatedly advised to stay in bed, keep the perineum clean, and maintain a reasonable diet, their various vital signs were monitored to closely observe for phenomena such as abdominal pain and vaginal bleeding, and in case of any abnormalities, the physicians were promptly informed for management; ② after admission, the patients' menstrual history and whether they had other severe systemic internal medicine diseases were carefully evaluated for identification and diagnosis; ③ the patients' vital signs were evaluated to judge the presence or absence of internal bleeding signs, and shock therapy (quickly establishing the vein passage, giving plenty of fluid and performing blood transfusion, monitoring various indicators such as blood pressure, heart rate, and body temperature, repeatedly warning the patients to keep a correct position to avoid condition progression, keeping the respiratory tract unobstructed, and performing oxygen inhalation when necessary) was applied for patients with shock signs; ④ physical intervention: before surgery, clinical intensive education in the form of face-to-face communication, individual guidance, etc., was carried out to enhance physical support and then eliminate patients' negative emotions as much as possible; the patients' emotions were kept stable before surgery so that they could actively accept the clinical treatment; ⑤ after surgery, patients' vital signs were closely observed, especially the volume of vaginal bleeding, incision pain, and infection signs, the patients were assisted to roll over and encouraged to do off-bed activities as soon as possible, the cleaning and nursing of the perineum were performed properly, and scientific dietary plans consisted of more foods with rich cellulose, vitamin, and protein were made; ⑥ medication guidance: the patients were repeatedly advised to take the medicine as directed and informed of the name, usage, dose, and precautions of the medicine to understand the adverse reactions and corresponding handling measures; ⑦ discharge guidance: the patients were guided to take reasonable birth control measures as directed, maintain good health habit to reduce the odds of pelvic infection, strengthen nutrition after surgery, and maintain sufficient sleep time, and regular follow-up was performed
2. Intelligent medical management platform. The patients were guided to log in to the “Intelligent medical management platform” app developed by our hospital, which contained three parts, i.e., health education, rehabilitation encyclopedia, and Q&A. Health education mainly included surgical process, key points of surgical cooperation, postoperative drug prescription, and dietary plan, the contents of each item were displayed in words, and some contents were presented with videos. Rehabilitation encyclopedia mainly introduced the prevention and handling measures for postoperative complications, including ① inflammatory reactions: in case of delayed wound healing due to wound infection, the patients' family members should closely observe the skin around the incision, and the patients were guided to orally take antibiotics for anti-infection as directed; ② pain: the patients were informed of possible extremity pain after surgery, and the nursing personnel or patients' family members could help the patients massage limbs or play relaxed and soothing music to relieve their pain sensation; ③ postoperative exercise: the patients were informed of the significance of avoiding strenuous exercise in the short term, forming good diet and exercise habits, and avoiding strong physical work during rehabilitation. In the Q&A part, patients' doubts were answered and physical therapy including willpower training, music therapy, intimation, and meditation was provided. The intervention time for the two groups was 30 d

RETRACTED

### 2.3. Observation Indicators

Cognition of disease. The nurses distributed the self-designed questionnaire on cognition of disease to each patient, which contained 10 items, including the cause of disease, clinical symptoms, postoperative precautions, and self-care methods. The hundred-mark system was applied to the questionnaire, with 95-100 points indicating complete cognition, 85-94 points indicating basic cognition, and <85 points indicating no cognition.

The degrees of satisfaction with clinical nursing of the two groups were evaluated by the questionnaire on patient satisfaction with nursing proposed by our hospital, with the evaluation items of psychological counseling, nursing operation, abnormal pain alleviation, and hospital management. The maximum score of each item was 100 points, and higher scores indicated higher satisfaction with nursing.

Patients' QOL was evaluated by the MOS item short-form health survey (SF-36) [13], which covered four aspects, i.e., social activities, physical activities, cognitive activities, and role activities. The maximum score of each item was 100 points, and higher scores indicated higher QOL.

RETRACTED

The occurrence of postoperative complications, including wound hemorrhage, abdominal distention, constipation, and retention of urine, was recorded and compared between the two groups.

### 2.4. Statistical Methods

The statistical software GraphPad Prism 7.0 was used for analysis, the measurement data were expressed by (mean ± SD), and the between-group comparisons were examined by *t*-test with independent samples; the enumeration data were expressed by (*n*(%)) and examined by the *X*^2^ test, and differences were considered statistically significant at *P* < 0.05.

## 3. Results

### 3.1. Between-Group Comparison of Baseline Data

Table 1 shows that no statistical between-group differences in the mean age, BMI values, type of disease, family economic situation, etc., were observed (*P* > 0.05), presenting the comparability.

### 3.2. Comparison of Cognitive Ability

Figure 1 shows that after intervention, the score on cognitive ability was significantly higher in EG than in RG (*P* < 0.001).

### 3.3. Comparison of Satisfaction with Nursing

Table 2 shows that after intervention, the scores on satisfaction with various nursing aspects were significantly higher in EG than in RG (*P* < 0.001).

### 3.4. Comparison of QOL Scores

Table 3 shows that after intervention, the scores on QOL were significantly higher in EG than in RG (*P* < 0.001).

### 3.5. Comparison of Occurrence of Complications

Table 4 shows that during the study, the total incidence rate of complications was significantly lower in EG than in RG (*P* < 0.05).

## 4. Discussion

Hysterectomy is a common gynecological surgical procedure, its surgical trauma is large, which can easily lead to postoperative stress incontinence, pelvic organ prolapse, insomnia, anxiety, and other problems in patients, adversely affecting patients' QOL and family function [14, 15]. In addition, surgery causes great psychological stress in patients, which, combined with the fact that patients have less knowledge about anesthesia and surgery, may trigger stress reactions and then have an impact on the circulation and neuroendocrine system, hindering the smooth implementation of surgery [16], so it is highly necessary to carry out clinical management during the perioperative period of hysterectomy. Routine nursing, although meeting the basic clinical needs of patients, is not comprehensive enough, and postoperative complications can still occur, affecting prognosis [17]. Detailed nursing has been widely used in the clinic in recent years, which, as a new type of proactive nursing model, can minimize the potential risks of surgery [18, 19]. Perioperative detailed nursing requires that nursing personnel carry out nursing according to the process, conduct each step strictly and normatively, and timely satisfy patients' needs, so it can help to improve the patients' clinical treatment compliance and promote early rehabilitation. After popularization, a detailed nursing model has been applied in liver cancer, nasal polyps, esophageal cancer, and other diseases [20].

RETRACTED

Nowadays, with the development of social science and technology, information technology is entering all walks of life in different ways, and likewise, intelligent medicine, a new type of medical service model, also appears in the medical industry [21] and has become a new target for the current development of medical and health careers. Studies found that [22] implementing necessary health education and management for patients in the perioperative period can accelerate the recovery of the condition and reduce the occurrence of complications. At present, traditional health education is mostly verbal preaching by nurses, and this one-way health knowledge delivery method is unfavorable for patients' understanding and mastery of disease-related knowledge. However, with the help of intelligent medical tools that are featured with easy reference and long-lasting preservation [23], patients can actively learn health education knowledge by watching the videos and understand their illness through the intelligent medical management platform, thereby avoiding nursing work emissions to some extent. In this study, the application value of the above-combined intervention was explored by implementing an intelligent medical management platform combined with perioperative detailed nursing for patients undergoing hysterectomy.

In terms of cognition of disease, the score on cognitive ability was significantly better in EG than in RG (*P* < 0.001), which might be due to the fact that the implementation of the intelligent medical management platform got rid of the traditional oral preaching mode, so that patients could learn the relevant knowledge of their own disease and have a comprehensive and detailed understanding of the disease etiology, surgical operations, postoperative precautions, dietary regimens, etc., which improved the effect of nursing implementation. In terms of the postoperative complications and QOL, the total incidence rate of complications during the study was significantly lower in EG than in RG (*P* < 0.05), and various scores on QOL were significantly higher in EG than in RG (*P* < 0.001), indicating that implementing intelligent medical management platform and detailed nursing could obviously improve the patients' QOL and lower the risk of triggering postoperative complications. The reasons may be that the intelligent medical management platform provides patients with a quality perioperative clinical management by integrating resources and realizing multidimension and all-round health education, Q&A, and other aspects to improve the patients' cognition of their own disease [24] and reduce the occurrence of complications and that with perioperative detailed nursing that covers many aspects, rational psychological nursing intervention is carried out to relieve the negative emotions of the patients and their family members and enhance their treatment confidence, and scientific dietary intervention is conducted to improve the body immunity and provide a guarantee for the postoperative rehabilitation, benefiting patients' recovery and prognosis [25].

RETRACTED

Limitation of the study: the questionnaire to evaluate patient satisfaction with nursing and the score on cognition of disease adopted in this study may bias the results. Therefore, greater research support is needed to ensure more safe and effective postoperative rehabilitation for patients undergoing hysterectomy and to improve the quality of medical nursing.

## 5. Conclusion

In conclusion, combining an intelligent medical management platform with perioperative detailed nursing for patients undergoing hysterectomy can significantly improve patients' satisfaction with clinical nursing and reduce the occurrence of complications, which is worthy of clinical reference.

## Figures and Tables

**Figure 1:** Comparison of cognitive ability (mean ± SD). Note: the horizontal axis indicated EG and RG, and the vertical axis indicated the cognitive ability score (points); the cognitive ability scores of EG and RG were, respectively, (81.84 ± 3.95) and (71.11 ± 3.57), and ∗ indicated a significant between-group difference in the cognitive ability scores (*t* = 12.423, *P* < 0.001).

**Table 1:** Between-group comparison of baseline data.

Item	EG	RG	*X* ^2^/*t*	*P*
Mean age (mean ± SD, years)	55.76 ± 5.32	55.68 ± 5.30	0.066	0.948
BMI (mean ± SD, kg/m^2^)	20.82 ± 0.98	20.53 ± 1.01	1.270	0.208
Surgery time (mean ± SD, min)	121.74 ± 6.94	121.55 ± 6.74	0.121	0.904
Type of disease				
Endometrial carcinoma	9 (23.68%)	11 (28.95%)	0.271	0.602
Uterus myoma	13 (34.21%)	10 (26.32%)	0.561	0.454
Adenomyosis	16 (42.11%)	17 (44.74%)	0.054	0.817
Family economic situation			0.211	0.646
≥3,000 yuan (month·person)	19 (50.00%)	21 (55.26%)		
<3,000 yuan (month·person)	19 (50.00%)	17 (44.74%)		
Place of residence (*n*(%))			3.378	0.066
Urban area	16 (42.11%)	14 (36.84%)		
Rural area	22 (57.89%)	24 (63.16%)		
Educational degree (*n*(%))				
Junior college and above	3 (7.89%)	4 (10.53%)	0.157	0.692
Senior high school	13 (34.21%)	11 (28.95%)	0.244	0.622
Junior high school and below	22 (57.89%)	23 (60.53%)	0.055	0.815

RETRACTED

**Table 2:** Between-group comparison of patient satisfaction with nursing after intervention (mean ± SD).

Group	*n*	Abnormal pain alleviation	Nursing operation	Hospital management	Psychological counseling
EG	38	82.34 ± 2.40	79.16 ± 2.38	77.18 ± 3.92	80.29 ± 3.84
RG	38	73.63 ± 3.77	68.26 ± 2.59	68.71 ± 2.59	67.66 ± 3.18
*t*		12.014	19.102	11.113	15.616
*P*		<0.001	<0.001	<0.001	<0.001

**Table 3:** Between-group comparison of QOL scores after intervention (mean ± SD).

Group	*n*	Role activities	Cognition activities	Social activities	Physical activities
EG	38	78.50 ± 4.06	80.50 ± 3.10	76.58 ± 3.92	80.53 ± 4.02
RG	38	70.58 ± 2.42	69.92 ± 3.98	69.34 ± 3.13	69.16 ± 3.51
*t*		10.329	12.928	8.897	13.133
*P*		<0.001	<0.001	<0.001	<0.001

**Table 4:** Between-group comparison of occurrence of complications (*n*(%)).

Group	*n*	Wound bleeding	Abdominal distension	Constipation	Retention of urine	Total incidence rate
EG	38	0 (0.00)	1 (2.63)	1 (2.63)	0 (0.00)	5.26% (2/38)
RG	38	2 (5.26)	3 (7.89)	2 (5.26)	1 (2.63)	21.05% (8/38)
*X* ^2^						4.146
*P*						<0.05

## Data Availability

The data to support the findings of this study is available on reasonable request from the corresponding author.
